The article "Comparison of 10-Year Survival Outcomes for Early Single Hepatocellular Carcinoma following Different Treatments" was retracted in 2023. Reasons: suspected computer-generated content; unreliable results or conclusions; concerns about the data; concerns about the results or conclusions.

# Comparison of 10-Year Survival Outcomes for Early Single Hepatocellular Carcinoma following Different Treatments

**DOI:** 10.1155/2021/6638117

**Published:** 2021-03-19

**Authors:** Fanyu Meng, Haoyun Zhang, Haiwen Peng, Shichun Lu

**Affiliations:** ^1^Department of Hepatobiliary Surgery, First Medical Center of Chinese People's Liberation Army (PLA) General Hospital, Beijing 100853, China; ^2^Department of Hepatobiliary Surgery, Chifeng Clinical Medical School of Inner Mongolia Medical University, Chifeng, Inner Mongolia 024000, China; ^3^Department of Orthopedics Surgery, First Medical Center of Chinese People's Liberation Army (PLA) General Hospital, Beijing 100853, China

## Abstract

**Introduction:**

To compare the actual 10-year survival outcomes of early single hepatocellular carcinoma (HCC) patients between 3 first-line treatments: radiofrequency ablation (RFA), surgical resection (SR), or transplantation (LT).

**Methods:**

A total of 1255 early single HCC patients retrieved from the Surveillance Epidemiology and End Results (SEER) database were included. Patients survived ≥10 years, and patients died <10 years were compared. Significant predictors associated with 10-year survival were identified by multivariate logistic regression analysis. The 10-year survival outcomes of 3 treatments were compared using multivariate model risk adjustment and inverse probability of treatment weighted (IPTW) adjustment.

**Results:**

Of the 1255 patients, 472 patients underwent SR, 259 patients underwent LT, and 524 patients underwent RFA. 149 patients achieved 10-year survival. Multivariate logistic regression analysis showed that age, race, treatment, and fibrosis score were significant predictors for 10-year survival, and LT had the best advantage of 10-year survival, followed by SR. Comparable 10-year survival outcomes were found between SR and RFA after IPTW. Then, a subgroup analysis was performed based on the tumor size, and the results showed that for ≤50 mm tumor, SR showed no significant advantages over RFA for 10-year survival.

**Conclusions:**

Estimates of the observational association of different treatments with 10-year survival are sensitive to the analytic method. LT showed the best outcomes for patients. No significant differences for 10-year survival were found between SR and RFA in the IPTW cohort. Subgroup analysis showed that for >50 mm tumor, SR showed significant advantages over RFA after IPTW.

## 1. Introduction

Hepatocellular carcinoma (HCC) is a common malignant tumor. It accounts for around 80% primary liver cancers worldwide [1]. HCC is estimated to be the fourth cause of cancer-related death overall worldwide [2]. Despite considerable progress in risk factor control, molecular profiles, early detection, diagnosis, treatment and so on, the incidence and cancer-related mortality in HCC patients are still increasing in many countries [3].

Several studies have focused on the 10-year survivors of HCC, and these studies only focus on one treatment [4–7]. Liver transplantation is the optimal treatment option for early HCC, but it was limited by lack of donor organs. One study reported that the actual 10-year survival rate for HCC patients who had liver transplantation was 41.1% [6]. For patients who underwent resection, the actual 10-year survival rate of patients was about 7.2%, whereas the actuarial survival quoted from the same studies was 26.8% [8]. Recurrence does not preclude long-term survival [9]. Different 10-year survival calculation methods lead to significant differences in results. The Kaplan-Meier method of actuarial survival analysis tends to overestimate survival outcomes [8]. Therefore, actual 10-year survivors were analyzed in this study.

Liver transplantation (LT), surgical resection (SR), and radiofrequency ablation (RFA) are recommended for early HCC [10]. The three treatments were all analyzed in this study. A total of 1255 early single HCC patients were included, and we overcame the limitation of small sample size and long-term follow-up using data from the SEER database. In order to better compare the effect of treatments on 10-year survival, we used IPTW, a propensity scoring method to minimize the treatment selection deviation. We identify patient characteristics associated with 10-year survival using multivariate logistic regression analysis. The 10-year survival outcomes of the 3 treatments were also compared.

## 2. Methods

### 2.1. Database and Patient Selection

The current study was a retrospective cohort study of HCC patients identified from the Surveillance Epidemiology and End Results (SEER) database. The data (incidence-SEER 18 Regs Custom Data with additional treatment fields, Nov 2018 Sub, 1975 -2016 varying) was obtained by the SEER^∗^Stat software (version 8.3.6; http://seer.cancer.gov/seerstat/). The following surgery codes were used: RFA : 16; SR : 20 to 25, 30, 36, 37, 50, 51, and 52; and LT : 61.

Patients with labeled primary sites of C22.0-liver and pathologically diagnosis (ICD-O-3 histologic type: 8170-8175) were carefully reviewed. The inclusion criteria were as follows: (1) first malignant tumor (*N* = 93230); (2) with detailed TNM stage information and no metastasis (*N* = 45655); (3) patients received RFA, SR, or LT were included (*N* = 11243); (4) single tumor (*N* = 7638); and (5) patients with at least 10-year follow-up were included, and patients who were alive but without 10-year follow-up were excluded (*N* = 3754). The exclusion criteria were as follows: (1) unknown race record (*N* = 10), (2) unknown exact tumor size (*N* = 137), and (3) unknown liver fibrosis score (*N* = 2352).

We collect sociodemographic data (age, sex, race), pathologic data (histologic type, grade, fibrosis score, tumor size, and *T* and *N* stages), and follow-up data for each patient. In the SEER database, the fibrosis score had been grouped into F0 (fibrosis score 0-4) and F1 (fibrosis score 5-6), respectively. Based on tumor size, tumor number, lymph node involvement, and vascular invasion, the AJCC 8^th^ edition staging systems were derived as previously reported [11].

### 2.2. Statistical Analyses

Descriptive statistics are reported as number of events, mean ± SD, or median (interquartile range). Differences between the 10-year survivors and 10-year nonsurvivors were compared using Student's *t*-test or Mann–Whitney *U* test for continuous variables. For categorical variables, chi-square test or Fisher exact test were performed. Then, univariate and multivariate logistic regression analysis was performed to identify independent predictive factors for 10-year survival. Propensity scores were estimated with multinomial logistic regression, with treatments as outcomes and age, sex, *T* stage, race, grade, tumor size, fibrosis score, and regional lymph node involvement as pretreatment covariates. Inverse probability of treatment weighted was calculated with the estimated propensity scores [12]. The standardized mean differences (SMD) in covariate values between treatment groups were compared in the IPTWs samples [13]. All statistical analysis was performed using *R* 3.6.1 (https://www.r-project.org/) and SPSS 22.0.

## 3. Results

### 3.1. Patient Characteristics

This study focused on the actual 10-year survival, so patients who were alive but without 10-year follow-up were excluded in this study. Finally, a total of 1255 patients who met the inclusion criteria were included in this study. The median follow-up of the whole cohort was 135 months for overall survival. 149 (11.87%) of them achieved 10-year survival. All patients had an early *T* stage; of them, 269 patients were at T1a stage, 828 patients were at T1b, and 158 were T2. Among them, 472 patients underwent liver resection, 259 patients underwent liver transplantation, and 524 patients underwent RFA. The actual 10-year survival rate of patients who underwent LT was 34.0%. For patients who underwent SR and RFA, the actual 10-year survival rate was 9.1% and 3.4%, respectively. As shown in Table 1, patients who survive ≥10 years were younger than those who survive <10 years. Besides, significant differences were also found in *T* stage (*P* = 0.021), race (*P* < 0.001), tumor grade (*P* = 0.011), and treatment (*P* < 0.001) between the two groups (Table 1). The survival curves of patients stratified by treatment were shown in Figure 1(a). The median survival months for RFA, SR, and LT were 24, 30, and 67 months, respectively.

### 3.2. Treatment Characteristics and Logistic Regression Analysis of Unadjusted Cohort

Patients' baseline characteristics stratified by treatment were shown in Table 2. The baseline characteristics comparison of the unweighted cohort showed that age (*P* < 0.001), *T* stage (*P* < 0.001), race (*P* < 0.001), grade (*P* < 0.001), tumor size (*P* < 0.001), and fibrosis score (*P* < 0.001) were significantly different among the 3 treatments. Only sex (*P* = 0.286) and regional lymph node involvement (*P* = 0.84) showed no significant differences among the 3 treatments and with the SMD less than 0.1. Multivariate logistic regression analysis adjusting for all baseline patient characteristics showed that age, race, treatment, and fibrosis score were significant predictors for 10-year survival as shown in Table 3. While sex, *T* stage, grade, tumor size, and regional lymph node involvement were not significant predictors for 10-year survival.

### 3.3. Patient and Treatment Characteristics of IPTW-Adjusted Cohort

IPTW was used to balance the patient baseline characteristics of the 3 treatments. After IPTW, only age, tumor size, and fibrosis score differed significantly between the 3 treatments as shown in Table 2. The survival curves of weighted cohort stratified by treatment were shown in Figure 1(b).The change of SMD is shown in Figure 1(c). After IPTW, the actual 10-year survival rate of patients who underwent LT, SR, and RFA was 33.1%, 8.4% and 3.8%, respectively. The univariate logistic regression analysis for 10-year survival was performed in the IPTW cohort, and the results were shown in Table 4 (model 3). The results showed that compared to RFA, patients who received LT have significant higher odds of 10-year survival (OR: 1.34, 95% CI: 1.25-1.45, *P* < 0.001), while patients who received SR had comparable odds of 10-year survival (OR: 1.05, 95% CI: 1.00-1.10, *P* = 0.066). IPTW cohort was further adjusted for age, tumor size, and fibrosis score in the multivariate logistic regression analysis, and the results showed that the 10-year survival odds for patients who received SR had no significant differences compared to RFA (OR: 1.04, 95% CI: 0.99-1.10, *P* = 0.138).

Unadjusted, multivariable adjusted, univariate IPTW-adjusted, and multivariable IPTW cohort logistic regression models for 10-year survival of the three treatments were shown in Table 4. Of the 4 methods used to compare 3 treatments, all showed that LT had the best advantage of 10-year survival compared to RFA, but the OR (95% CI) of the LT vs RFA decreased from 14.47 (8.66-25.44) in the model 1 to 1.34 (1.24-1.45) in the model 4. Similar results shown in SR vs RFA. These results suggested the presence of treatment selection bias. Moreover, after IPTW, patients who underwent RFA showed comparable 10-year survival with SR as shown in Table 4 (model 3 and model 4).

### 3.4. Subgroup Analysis

Although RFA showed comparable 10-year outcomes with SR in the entire IPWT cohort, the therapeutic effect of RFA is affected by the tumor size, of which the most commonly reported size cutoff values are 30 mm and 50 mm [14, 15]. Therefore, we stratified patients into different tumor size groups according to 30 mm and 50 mm. Then, after reweighting by IPTW, the 10-year survival outcomes were compared in each group. As shown in Table 5, for ≤30 mm tumor, LT showed significant advantages over SR (*P* < 0.001) and RFA (*P* < 0.001), but no significant differences were found between SR and RFA. For 30-50 mm tumor, only the comparison between LT and RFA showed significant differences, while no significant differences were found for SR vs RFA (*P* = 0.090) and LT vs SR (*P* = 0.192). For >50 mm tumor, LT showed the best outcomes, followed by SR.

## 4. Discussion

In this study, 1255 HCC patients with early and very early stage were included in this study. Univariate and multivariate logistic regression analysis was used to compare the actual 10-year survival outcomes of 3 treatments for HCC patients. IPTW was used to balance the bias between 3 treatments.

Using multivariate logistic regression analysis adjusted for patient covariates, the significant predictors for 10-year survival of early-stage HCC were age, race, treatment, and fibrosis score. However, *T* stage and tumor size were not significant predictors for the early single HCC. Among these predictive factors, fibrosis score is an important one. Cirrhosis was reported to be an independent risk factor associated with actual 10-year survival after hepatectomy of HBV-related HCC [4]. In this study, we found that patients with high fibrosis score (OR 0.58, 95% CI: 0.36-0.92) were associated with less chance of l0-year survival compared with those who had low fibrosis score in the multivariate logistic regression analysis.

The comparisons of the outcomes between different treatments may be biased due to important baselines differences among patients, often as a result of treatment selection biases [16]. Therefore, to efficiently reduce the effect of treatment selection bias, IPTW was used in this study. IPTW effectively reduces the bias of baseline characteristics among treatment modalities as shown in Figure 1(c). After IPTW, the OR for 10-year survival of LT vs RFA decreased from 14.47 (95% CI: 8.66-25.44) in the model 1 to 1.34 (95% CI: 1.24-1.45) in the model 4 for early single nodule HCC patients. These results suggested that the estimation of the observational association between different treatments and 10-year HCC survival is highly sensitive to the analysis method. In each model, LT still showed the significant best survival advantage over other treatments. SR (OR:2.22, 95% CI: 1.15-4.39, *P* = 0.019) showed significant differences with RFA in the multivariate logistic regression model of the unadjusted cohort, while SR (OR: 1.04,95% CI: 0.99-1.10, *P* = 0.138) showed no significant differences with RFA in the IPTW cohort (model 4).

Only 20% of HCC patients are eligible for surgical resection [17]. Many HCC patients are not suitable for surgery due to long-term virus infection, impaired liver function, fibrosis, tumor location, and multifocal tumors. Therefore, more patients are candidates for curative therapy with RFA. Although RFA was often used in patients who were ineligible for SR, we found that for early single tumor, patients who underwent RFA showed comparable 10-year survival outcomes with SR. Similarly, one study reported that RFA could achieve long-term survival for as long as 10 years [7]. RFA can provide similar long-term survival results to SR of single nodular HCC when combined with multimodal treatment [18]. These results support RFA as first-line treatment for early HCC, especially for patients with ≤50 mm tumor as shown in the subgroup analysis (Table 5). Moreover, RFA is a safe treatment. Complications occurred in only 2.2% of the treatments [7]. Another study reported that the complication rate was 1.8% [19].

Although comparable outcomes between RFA and SR for small tumors (≤3 cm), RFA is associated with higher rates of tumor recurrence and local disease progression, and the median 3- and 5-year survival rates were lower in this group [14]. In this study, the actual 10-year survival rate of SR (9.1%) was higher than RFA (3.4%). After IPTW, patients who underwent SR also showed better survival outcomes. The actual 10-year survival rate of SR and RFA was 8.4% and 3.8%, respectively. Therefore, surgical resection was still the preferred choice.

There are some limitations in this work. First, the variables supplied in the SEER databases were limited, and we could not get more detailed patient information like hepatitis and tumor location. Second, the database does not supply the actual fibrosis score, fibrosis score 0–4 means none to moderate fibrosis, and fibrosis score 5–6 means severe fibrosis or cirrhosis. Third, the database did not collect information on recurrence; thus, the impact of disease recurrence on patients' long-term survival could not be assessed. Fourth, the survival data was not restricted to cancer-related death; thus, patients in this study may die for other reasons.

Estimation of the observational link between different treatments and 10-year survival is sensitive to analytical methods. LT was the best treatment for early single HCC. Due to shortage of donors, SR and RFA both serve as effective treatments. No significant differences for 10-year survival were found between SR and RFA in the IPTW cohort especially for ≤50 mm tumor.

## Figures and Tables

**Figure 1:** Overall survival of patients stratified by treatment (a). Overall survival of inverse probability treatment weighted-adjusted cohort stratified by treatment (b). Comparison of baseline characteristic standardized mean differences (SMD) of patients before and after inverse probability treatment weighting (c).

**Table 1:** Comparison of patient characteristics between 10-year survivors and 10-year nonsurvivors.

Variables	<10 year	≥10 year	*P*
	(*N* = 1106)	(*N* = 149)	
Age (mean (SD))	62.33 (9.75)	55.94 (10.22)	<0.001
Sex (%)			0.91
Male	855 (77.3)	114 (76.5)	
Female	251(22.7)	35(23.5)	
*T* stage (%)			0.021
T1a	224 (20.3)	45 (30.2)	
T1b	740 (66.9)	88 (59.1)	
T2	142 (12.8)	16 (10.7)	
Race (%)			<0.001
Black	136 (12.3)	4 (2.7)	
Other	264 (23.9)	52 (34.9)	
White	706 (63.8)	93 (62.4)	
Grade (%)			0.011
Well differentiated	200 (18.1)	37 (24.8)	
Moderately differentiated	361 (32.6)	59 (39.6)	
Poorly differentiated	138 (12.5)	17 (11.4)	
Unknown	407 (36.8)	36 (24.2)	
Tumor size (median (interquartile range))	32 (23-48)	30 (20-45)	0.044
Fibrosis score (%)			0.432
F0	332(30)	50 (33.6)	
F1	774 (70.0)	99 (66.4)	
Regional lymph node involvement (%)			0.335
No	1097 (99.2)	146 (98.0)	
Yes	9 (0.8)	3 (2.0)	
Therapy (%)			<0.001
RFA	506 (45.8)	18 (12.1)	
Resection	429 (38.8)	43 (28.9)	
Liver transplantation	171 (15.4)	88 (59.0)	

**Table 2:** Baseline characteristics of patients undergoing radiofrequency ablation, surgical resection, or liver transplantation in the unweighted and weighted study population.

	Unweighted cohort					Weighted cohort				
	Resection	Live transplantation	RFA	P	SMD	Resection	Live transplantation	RFA	P	SMD
	472	259	524			1060.73	934	1080.03		
Age (mean (SD))	62.79 (11.23)	56.85 (7.42)	62.80 (9.27)	<0.001	0.445	61.64 (10.38)	59.38 (7.74)	61.99 (9.19)	0.005	0.196
Sex = male (%)	355 (75.2)	208 (80.3)	406 (77.5)	0.286	0.082	806.7 (76.1)	737.1 (78.9)	830.5 (76.9)	0.778	0.046
*T* stage (%)				<0.001	0.588				0.531	0.122
T1a	47 (10.0)	94 (36.3)	128 (24.4)			206.1 (19.4)	220.3 (23.6)	238.6 (22.1)		
T1b	312 (66.1)	141 (54.4)	375 (71.6)			706.1 (66.6)	607.9 (65.1)	743.0 (68.8)		
T2	113 (23.9)	24 (9.3)	21 (4.0)			148.5 (14.0)	105.9 (11.3)	98.5 (9.1)		
Race (%)				<0.001	0.345				0.651	0.106
Black	58 (12.3)	17 (6.6)	65 (12.4)			117.5 (11.1)	92.2 (9.9)	116.6 (10.8)		
Other	158 (33.5)	42 (16.2)	116 (22.1)			292.0 (27.5)	200.3 (21.4)	260.4 (24.1)		
White	256 (54.2)	200 (77.2)	343 (65.5)			651.1 (61.4)	641.5 (68.7)	703.1 (65.1)		
Grade (%)				<0.001	0.956				0.108	0.212
Well differentiated	86 (18.2)	64 (24.7)	87 (16.6)			211.4 (19.9)	175.8 (18.8)	207.6 (19.2)		
Moderately differentiated	245 (51.9)	96 (37.1)	79 (15.1)			400.3 (37.7)	307.6 (32.9)	348.4 (32.3)		
Poorly differentiated	98 (20.8)	32 (12.4)	25 (4.8)			153.4 (14.5)	108.2 (11.6)	86.2 (8.0)		
Unknown	43 (9.1)	67 (25.9)	333 (63.5)			295.6 (27.9)	342.4 (36.7)	437.7 (40.5)		
Tumor size (mean (SD))	58.29 (43.14)	27.86 (14.33)	31.13 (14.85)	<0.001	0.671	42.99 (34.07)	32.49 (15.33)	34.86 (19.15)	<0.001	0.276
Fibrosis score = F1 (%)	225 (47.7)	221 (85.3)	427 (81.5)	<0.001	0.576	701.0 (66.1)	726.3 (77.8)	813.2 (75.3)	0.021	0.174
Lymph node involvement = yes (%)	4 (0.8)	2 (0.8)	6 (1.1)	0.84	0.026	7.3 (0.7)	4.1 (0.4)	15.3 (1.4)	0.28	0.069

**Table 3:** Univariate and multivariate logistic regression analysis of predictors for 10-year survival in all patients (unweighted cohort).

Variable	Univariate		Multivariate	
	OR (95% CI)	*P*	OR (95% CI)	*P*
Age, year	0.94 [0.92-0.95]	<0.001	0.95 [0.93-0.97]	<0.001
Sex (male vs female)	0.96 [0.64-1.45]	0.828	0.77 [0.49-1.22]	0.255
Race				
Black	1		1	
Other	6.70 [2.67-22.48]	<0.001	7.70 [2.90-26.82]	<0.001
White	4.48 [1.83-14.82]	0.004	3.71 [1.45-12.62]	0.015
*T* stage				
T1a	1			
T1b	0.59 [0.40-0.88]	0.008	0.99 [0.60-1.63]	0.957
T2	0.56 [0.30-1.01]	0.062	0.76 [0.35-1.59]	0.471
Grade				
Well differentiated	1		1	
Moderately differentiated	0.88 [0.57-1.39]	0.586	0.85 [0.51-1.42]	0.526
Poorly differentiated	0.67 [0.35-1.21]	0.194	0.61 [0.29-1.24]	0.180
Unknown	0.48 [0.29-0.78]	0.003	0.74 [0.42-1.31]	0.611
Tumor size, mm	0.99 [0.99-1.00]	0.065	1.00 [0.99-1.00]	0.496
Treatment				
RFA	1		1	
Resection	2.82 [1.63-5.07]	<0.001	2.22 [1.15-4.39]	0.019
Liver transplantation	14.47 [8.66-25.44]	<0.001	12.62 [7.22-23.12]	<0.001
Fibrosis score (F1 vs F0)	0.85 [0.59-1.23]	0.379	0.58 [0.36-0.92]	0.02
Regional lymph node involvement (yes vs no)	2.50 [0.55-8.50]	0.172	2.08 [0.39-8.89]	0.345

**Table 4:** Association of treatments and 10-year survival among HCC patients using different analytic models.

Models	OR (95% CI)	*P* value
Univariate logistic regression model of the unadjusted cohort (model 1)		
LT vs RFA	14.47 [8.66-25.44]	<0.001
SR vs RFA	2.82 [1.63-5.07]	<0.001
LT vs SR	5.13 [3.44-7.76]	<0.001
Multivariable logistic regression model of the unadjusted cohort (model 2)		
LT vs RFA	12.62 [7.22-23.12]	<0.001
SR vs RFA	2.22 [1.15-4.39]	0.019
LT vs SR	5.69 [3.38-9.80]	<0.001
IPTW-adjusted (model 3)		
LT vs RFA	1.34 [1.25-1.45]	<0.001
SR vs RFA	1.05 [1.00-1.10]	0.066
LT vs SR	1.28 [1.18-1.40]	<0.001
IPTW and adjusted for age, tumor size, and fibrosis score (model 4)		
LT vs RFA	1.34 [1.24-1.45]	<0.001
SR vs RFA	1.04 [0.99-1.10]	0.138
LT vs SR	1.28 [1.17-1.41]	<0.001

**Table 5:** Subgroup analysis according to the tumor size for 10-year survival outcomes between 3 treatments after reweighting by IPTW in each group.

Tumor size	Number of patients	Actual 10-year survival outcome		
		LT vs RFA	SR vs RFA	LT vs SR
≤30	613	1.35 [1.24-1.48] *P* < 0.001	1.00 [0.97-1.04] *P* = 0.796	1.35 [1.23-1.47] *P* < 0.001
30-50	378	1.25 [1.10-1.42] *P* = 0.001	1.12 [0.98-1.27] *P* = 0.090	1.12 [0.94-1.33] *P* = 0.192
>50	264	1.54 [1.14-2.07] *P* = 0.005	1.08 [1.03-1.13] *P* = 0.001	1.42 [1.05-1.91] *P* = 0.022

## Data Availability

The analyzed data are available from the corresponding author on reasonable request.
